This article has been retracted.

# Inhibition of Spontaneous Recovery of Fear by mGluR5 after Prolonged Extinction Training

**DOI:** 10.1371/journal.pone.0059580

**Published:** 2013-03-21

**Authors:** Sheng-Chun Mao, Chih-Hua Chang, Chia-Chen Wu, Maria Juliana Orejanera, Olivier J. Manzoni, Po-Wu Gean

**Affiliations:** 1 Institute of Basic Medical Sciences and Department of Pharmacology, National Cheng-Kung University, Tainan, Taiwan; 2 INSERM U901, Marseille, France; Western University of Health Sciences, United States of America

## Abstract

Fear behavior is vital for survival and involves learning contingent associations of non-threatening cues with aversive stimuli. In contrast, excessive levels of fear can be maladaptive and lead to anxiety disorders. Generally, extensive sessions of extinction training correlates with reduced spontaneous recovery. The molecular mechanisms underlying the long-term inhibition of fear recovery following repeated extinction training are not fully understood. Here we show that in rats, prolonged extinction training causes greater reduction in both fear-potentiated startle and spontaneous recovery. This effect was specifically blocked by metabotropic glutamate receptor 5 (mGluR5), but not by mGluR1 antagonists and by a protein synthesis inhibitor. Similar inhibition of memory recovery following prolonged extinction training was also observed in mice. In agreement with the instrumental role of mGluR5 in the prolonged inhibition of fear recovery, we found that FMR1−/− mice which exhibit enhanced mGluR5-mediated signaling exhibit lower spontaneous recovery of fear after extinction training than wild-type littermates. At the molecular level, we discovered that prolonged extinction training reversed the fear conditioning-induced increase in surface expression of GluR1, AMPA/NMDA ratio, postsynaptic density-95 (PSD-95) and synapse-associated protein-97 (SAP97). Accordingly, delivery of Tat-GluR2_3Y_, a synthetic peptide that blocks AMPA receptor endocytosis, inhibited prolonged extinction training-induced inhibition of fear recovery. Together, our results demonstrate that prolonged extinction training results in the mGluR5-dependent long-term inhibition of fear recovery. This effect may involve the degradation of original memory and may explain the beneficial effects of prolonged exposure therapy for the treatment of phobias.

## Introduction

Fear behavior involves the contingent associations of non-threatening cues with aversive stimuli. Although necessary to survival, excessive levels of fear can be maladaptive and lead to anxiety disorders.

A commonly used protocol referred to extinction training is to repeatedly present non-threatening cues (conditioned stimulus, CS) to the subject without pairing with aversive stimuli (unconditioned stimulus, US) which results in a gradual decrease in conditioned response (CR) [1], [2]. This extinction process represents an explicit model of behavioral therapy and is an effective treatment for anxiety disorders including phobias and post-traumatic stress disorder [3]. Unfortunately, extinction is a new inhibitory learning that inhibits expression of the original association rather than its erasure [4]–[7] and reduction of fear through behavioral therapy is often followed by a return of fear. This idea is supported by a variety of experimental maneuvers that cause fear return including changing the test context (renewal) [8], presenting unsigned US (reinstatement) [9], or simply allowing time to pass (spontaneous recovery) [10].

Previous studies have shown that long-term potentiation (LTP) of synapses from auditory thalamus and cortex to the lateral amygdala (LA) is a key molecular event leading to the encoding of fear memory [11], [12]. Fear conditioning drives the synaptic insertion of AMPA receptors in the amygdala [13]. Indeed, by labeling surface receptors with biotin or using membrane fractionation approaches, we have reported that fear conditioning resulted in an increase in surface expression of GluR1 subunit of AMPA receptors in the amygdala [14]. More recently, we also found that 3 sessions of 10 presentations of light-alone trials applied 24 h after training reduced fear-potentiated startle without influencing the conditioning-induced increase in surface GluR1 [15]. Consistent with previous reports, the extinguished rats exhibited reinstatement and spontaneous recovery of fear.

Extinction of fear often takes more trials than acquisition and once initiated further CS presentations are more effective with spaced than with massed CS presentations [16]. To investigate the mechanisms underlying extinction, we apply two to eight sessions of 15 presentations of light-alone trials to test their effects on fear-potentiated startle, spontaneous recovery and conditioning-induced increase in surface GluR1.

## Results

### Recovery of Fear after Extinction Training Depends on the Number of CS-alone Trials

We have previously shown how rats that had received 30 CS-alone trials 24 h after training exhibited spontaneous recovery and reinstatement of fear [15]. Here we tested whether increasing the number of extinction trials could prevent spontaneous recovery and thus result in a more enduring reduction in fear responses. To that end, we randomly divided rats into 8 groups after 10 light-shock pairings. Groups 1–7 were given extinction training consisting of 2–8 sessions of 15 presentations of light-alone trials respectively and the percentage of fear-potentiated startle was measured 24 h after trials (Day 3, Test 1). The 8^th^ group was exposed to the context at equivalent time without receiving light-alone trials (context control group). Figure 1A shows that light-alone trial resulted in a reduction in startle potentiation. Startle potentiation were 201.2±19.2% (n = 7) in context controls, 74.4±11.4% (CS30, n = 7), 60.1±10.0% (CS45, n = 7), 53.0±10.4% (CS60, n = 7), 47.2±10.9% (CS75, n = 7), 41.6±6.7% (CS90, n = 7), 38.0±11.8% (CS105, n = 7) and 43.4±10.4% (CS120, n = 7) in extinction animals. The ANOVA for startle scores showed a significant effect for group (F_(7,48)_ = 24.61, *p*<0.001). In addition, less startle reflex occurred in the CS90, CS105 and CS120 groups than in the CS30 group (*p*<0.05), indicating that the effect depended on the number of CS-alone trials.

**Figure 1:** Recovery of fear after extinction training depends on the number of CS-alone trials. (A) Plot of percent startle potentiation in context control and extinction rats. Rats received 10 light-shock pairings and were randomly assigned to 2 to 8 sessions of extinction training groups. Rats in 2 or 8 sessions of extinction groups received 2 or 8 sessions of 15 presentations of light-alone trials without footshock and memory retention was assessed 24 h later (Test 1). Context control rats were returned to the startle box at the equivalent time without receiving light-alone trials. All groups were also tested on day 8 (Test 2) and Day 15 (Test 3). ***p<0.001, **p<0.01, *p<0.05 vs. context controls. (B) Inhibition of spontaneous recovery by prolonged extinction training is blocked by mGluR5 antagonist. MTEP was administered intraperitoneally (2.5, 5 or 10 mg/kg) 60 min before light-alone trials or was infused into the amygdala (10 µg/per side) abilaterally 30 min before CS-alone trials. ***p<0.001, *p<0.05 vs. saline. (C) Distribution of cannula tips in the amygdala from rats infused with MTEP (10 µg/per side) in experiments B. (D) MTEP was without effect on the 30 CS-alone trials-induced extinction memory. (E) Distribution of cannula tips in the amygdala from rats infused with MTEP (10 µg/per side) in experiments D. (F) CPCCOEt (5 or 10 mg/kg) injected intraperitoneally 60 min before light-alone trials failed to affect 90 CS-induced extinction of fear memory.

To determine whether the fear response could spontaneously recover some time after extinction training, all groups were also tested on day 8 (Test 2) and day 15 (Test 3) and their fear-potentiated startles were compared with their respective Test 1. As shown in figure 1A, fear responses were markedly reduced in animals receiving 90, 105 and 120 CS-alone trials. One-way ANOVA revealed a significant effect of groups among Test 2 (F_(7,48)_ = 10.69, *p*<0.001) and Test 3 (F_(7,48)_ = 9.97, *p*<0.001). Looking at each group individually we first found that the CS30, CS45, CS60 and CS75 groups showed increased startle potentiation (spontaneous recovery) in Test 3 relative to Test 1. On the other hand, CS90, CS105 and CS120 groups did not. Such absence of spontaneous recovery did not reflect a passive loss of fear memory because context control rats retained a stable memory for 14 days.

These results suggest that spontaneous recovery of fear after extinction can be retarded if sufficient CS-alone trials are delivered. Since little spontaneous recovery occurred after 90, 105 or 120 CS trials, 90 CS trials were used in the following experiments to elucidate the underlying mechanisms.

### mGluR5 Drive the Inhibition of Spontaneous Fear Recovery after Prolonged Extinction Training

A series of experiments were conducted to identify the receptor that mediated prolonged extinction training. Activation of group 1 metabotropic glutamate receptors (mGluRs) induce a distinct form of long-term depression (LTD) attributable to the endocytosis and decreased surface expression of postsynaptic AMPARs [17]–[19]. To test the possible involvement of group 1 mGluRs, we examined the effect of 3-[(2-methyl-1,3-thiazol-4-yl)ethynyl]pyridine (MTEP), a non-competitive antagonist of mGluR5 [20], [21] on prolonged extinction training. Rats were conditioned with 10 light-shock pairings and 24 h later received 6 sessions of 15 presentations of light-alone trials. MTEP was administered intraperitoneally (2.5, 5 or 10 mg/kg) 60 min before light-alone trials. These doses of MTEP have been shown to impair auditory fear conditioning [22]. Fear-potentiated startles were measured at 2, 7 and 14 days after conditioning. The results showed a significant effect for group (F_(3,24)_ = 17.85, *p*<0.001), and Newman-Keuls *post hoc* tests revealed that the level of startle potentiation in the 5 and 10 mg/kg rats was significantly higher than that of the 2.5 mg/kg rats (*p*<0.001) indicating a dose-dependent effect. There were no differences between saline and 2.5 mg/kg MTEP for Test 2 and Test 3 (*P*>0.1). Furthermore, the levels of startle potentiation in the 5 and 10 mg/kg rats were equivalent to the levels observed in rats conditioned without light (*p*>0.05) (Fig. 1B). These results suggest that systemic application of MTEP before CS-alone trials attenuated inhibition of spontaneous recovery of fear memory. Similar to systemic administration, direct infusion of MTEP (10 µg/side, n = 7) into the amygdala 30 min before light-alone trials attenuated inhibition of fear recovery, demonstrating the key role of amygdala mGluR5 in this effect.

To examine whether mGluR5 was involved in the effect of 30 CS-alone trials, we repeated the experiments except that 90 CS-alone trials were replaced by 30 CS-alone trials. Comparison among 30 CS-alone (no drug treatment) and two MTEP groups revealed no significant differences on Test 1 (F_(2,18)_ = 0.105, n = 7 in each group, *p*>0.5), Test 2 (F_(2,18)_ = 0.129, *p*>0.5) and Test 3 (F_(2,18)_ = 0.181, *p*>0.5) in these 3 groups. Thus, in contrast to 90 CS-alone trials, mGluR5 is not involved in 30 CS-alone extinction memory.

To exclude a contribution of mGluR1, we evaluated the effect of mGluR1 receptor selective antagonists [7-(hydroxyimino)cyclopropa[b] chromen-1a-carboxylate ethyl ester (CPCCOEt) [23] on extinction. CPCCOEt (5 or 10 mg/kg, i.p.), at the doses reported to induce central effects [24], had no effect on the 90 CS-alone-induced extinction (Fig. 1F). Together results suggest that mGluR5 but not mGluR1 receptor is involved in the extensive extinction training-induced extinction of fear memory.

### mGluR5-dependent Inhibition of Fear Recovery Requires Protein Synthesis

Induction of LTD by group 1 metabotropic glutamate receptor required rapid dendritic protein synthesis [25], [26]. Thus, we determined the effect of a potent protein synthesis inhibitor on extinction. Anisomycin was administered intraperitoneally (100 mg/kg) 60 min before light-alone trials. One-way ANOVA of startle amplitude for vehicle, anisomycin and context control rats indicated a main effect of group (F_(2,18)_ = 41.18, *p*<0.001) with anisomycin rats showing significantly higher startle amplitude than that of vehicle-treated rats (*p*<0.001) and equivalent startle amplitude to context control rats (*p*>0.05) (Fig. 2A). Similarly, intra-amygdala application of anisomycin (62.5 µg/side, n = 7) 30 min before light-alone trials blocked extinction (F_(2,18)_ = 29.69, *p*<0.001).

**Figure 2:** Protein synthesis is required for 90 CS-alone trials-induced inhibition of spontaneous recovery. (A) Rats were conditioned with 10 light-shock pairings and 24 h later received 6 sessions of 15 presentations of light-alone trials. Anisomycin was administered intraperitoneally (100 mg/kg, n = 7) 60 min before light-alone trials or was infused into the amygdala (62.5 µg/side, n = 7) 30 min before light-alone trials. ***p<0.001 vs. vehicle. (B) Distribution of cannula tips in the amygdala from rats infused with Anisomycin (62.5 µg/side, n = 7).

### Contextual Fear Conditioning and Prolonged Extinction in Wild Type and FMR1^−/−^ Mice

To extend our previous observation in rats, we reproduced our main results in mice. Mice were placed in a context for 3 min and received a footshock every 60 sec for 5 times. After training, mice were randomly assigned to saline, 2.5 mg or 5 mg MTEP groups. As shown in figure 3A, all experimental groups acquired equivalent amount of conditioned freezing. On day 2, mice were placed in the same context for 10 min without receiving footshock. The procedure was repeated 3 times with interval of 30 min (Extinction training). Contextual freezing responses were measured on day 3 and day 8. Figure 3A shows that all groups exhibited a similar decrement of freezing. The effect of drug was not significant at the last min of extinction training on day 2 (F_(2, 27)_ = 0.021, *p>*0.5). However, on day 3 and day 8, mice of pre-extinction injection of MTEP 5 mg/kg showed higher level of freezing compared with saline and MTEP 2.5 mg/kg groups (Day 3: F_(2, 27)_ = 4.45, *p<*0.05; Day 8: F_(2, 27)_ = 4.90, *p<*0.05). In addition, intraperitoneal injection of CPCCOEt (10 mg/kg) to mice before extinction training did not affect contextual freezing in both day 3 (T_(18)_ = 0.35, *p*>0.5 vs. vehicle) and day 8 (T_(18)_ = 0.54, *p*>0.5 vs. vehicle) (Fig. 3B). These results suggest that mGluR5 also is involved in the inhibition of spontaneous fear recovery after prolonged extinction training in mice.

**Figure 3:** Effects of mGluR5 antagonist and protein synthesis inhibitor on prolonged extinction training-induced inhibition of spontaneous recovery in mice. (A) On day 1, mice were placed in a context for 3 min and received a footshock every 60 sec for 5 times. On day 2, mice received intraperitoneal injection of saline, 2.5 mg/kg or 5 mg/kg of MTEP and 60 min later they were placed in the same context for 10 min without receiving footshock (extinction training). The extinction training was repeated 3 times with an interval of 30 min. Contextual freezing responses were measured as an index for memory retention on day 3 and day 8. *p<0.05 vs. saline or MTEP 2.5 mg. (B) CPCCOEt (10 mg/kg) injected intraperitoneally 60 min before extinction training failed to affect 90 CS-induced extinction of fear memory. (C) Same experimental procedure as (A) except anisomycin (62.5 µg/side, n = 10) or vehicle (n = 10) was infused into the hippocampus bilaterally 30 min before extinction training. *p<0.05 vs. vehicle. (D) Distribution of cannula tips in the hippocampus from mice infused with Anisomycin (62.5 µg/side, n = 10) or vehicle (n = 10).

We also determined the effect of protein synthesis inhibitor on extinction in mice. Since contextual fear memory is thought to depend upon the hippocampus [27], anisomycin was injected bilaterally into the hippocampus. Figure 3C shows that mice that had received intra-hippocampal injection of anisomycin (62.5 µg/per side, n = 10) before extinction training exhibited higher levels of freezing on both day 3 (T_(18)_ = 2.98, *p*<0.01 vs. vehicle) and day 8 (T_(18)_ = 2.67, *p<0.05* vs. vehicle). These results suggest that protein synthesis is required for the inhibition of fear memory recovery.

Genetic deletion of fragile X mental retardation protein (FMRP) is generally linked to the enhancement of mGluR5 signaling and dendritic protein synthesis-dependent mGluR long-term depression (mGluR-LTD) is upregulated in FMR1^−/−^ mice [26], [28]. To confirm our hypothesis of a key role of mGluR5 in fear memory recovery, we examined whether extinction training was altered in FMR1^−/−^ mice. Acquisition and extinction of contextual fear conditioning in FMR1^−/−^ mice (n = 8) and WT littermates (n = 7) are shown on figure 4. At the end of the acquisition session both genotypes exhibited similar levels of freezing behavior. Two-way repeated measures ANOVA (time x genotype) revealed a non-significant main effect of genotype [F_(1, 13)_ = 0.348, *p*>0.05] and a significant main effect of time [F_(7,91) = _41.577, *p*<0.001] (Fig. 4A). On day 2, mice underwent three 10 min extinction sessions in the conditioning context. FMR1^−/−^ mice showed decreased freezing levels from minute one to ten indicating both impaired fear conditioning and increased rate of extinction [F_(1,13) = _21.277, *p*<0.001]. Lower freezing levels were maintained in FMR1^−/−^ mice compared to WT animals in subsequent extinction sessions, two [F_(1,13) = _33.394, *p*<0.001] and three [F_(1,14) = _8.242, *p*<0.05] (Fig. 4B, C, D), showing that inhibitory learning was increased in FMR1^−/−^ mice. This effect was maintained in time as revealed by lower freezing levels on day 3 [F_(1,14) = _6.251, *p*<0.05] and 8 [F_(1,14) = _16.052, *p*<0.01] after conditioning (Fig. 4E). These results are compatible with our working hypothesis that mGluR5 are instrumental to fear recovery.

**Figure 4:** Contextual fear conditioning and extinction in FMR1−/− mice and WT littermates. (A) Acquisition of contextual fear conditioning. Mice were placed in a context for 3 min and received a foot shock every 60 sec for 5 times. Mice significantly increase freezing responses when compared to baseline (BL) measures before US presentation **p<0.01; ***p<0.001 *vs.* baseline (pairwise comparison test). (B) Extinction training. Mice underwent 3 extinction sessions with and interval of 30 min on day 2. *p<0.05; **p<0.01; ***p<0.001 (genotype effect). (C) Retention test. Freezing behavior was measured on day 3 and day 8 to evaluate long-term extinction memory *p<0.05; **p<0.01 (genotype effect). Data are expressed as mean ±s.e.m.

### Reversal of Conditioning-induced GluR1 Expression by 90 CS-alone Trials

We have previously shown that fear conditioning elicited an increase in surface expression of GluR1 subunit of AMPA receptors in the amygdala which was unaffected by 30 CS-alone trials [15]. Thus, we evaluated whether 90 CS-alone trials produced differential action on the conditioning-induced GluR1 expression. Rats were conditioned and 24 h later received 2–6 sessions of light-alone trials. Twenty-four hours later, LA and Basolateral Amygdala (BLA) tissues were dissected out and surface receptors were labeled with biotin. Biotinylated receptors were precipitated and surface GluR1 was determined by immunoblotting. Figure 5A shows that conditioning-induced increase in GluR1 was absent after 6 sessions of light-alone trials but was not affected by 2–4 sessions of trials (F_(5,30)_ = 7.36, *p*<0.001). Similarly, 90 CS-alone trials reversed conditioning-induced increase in GluR2 (F_(5,30)_ = 5.91, *p*<0.001) (Fig. 5A, right).

**Figure 5:** Reversal of conditioning-induced increases in surface expression of GluR1 and GluR2 is mediated by mGluR5. (A) Representative blots and mean ± SEM of GluR1 (left) and GluR2 (right) immunoreactivities from rats that had been conditioned with 10 light-shock pairings and 24 h later received 2–6 sessions of 15 presentations of light-alone trials. Lateral (LA) and basolateral (BLA) amygdala tissues were dissected out, and surface GluR1 and GluR2 levels were determined by biotin labeling. **p<0.01, *p<0.05 vs. context control. (B) GluR1 and GluR2 surface levels were normalized to total protein in the left, and GluR1 and GluR2 intracellular levels were normalized to total protein in the right. Conditioning-induced increase in GluR1 and GluR2 surface levels and decrease in GluR1 and GluR2 intracellular levels were reversed after 90 CS-alone trials (CS). The effect of 90 CS-alone trials was blocked in a dose dependent manner by MTEP (2.5–10 mg/kg, i.p.) or by intra-amygdala infusion of MTEP (10 µg/side). ***p<0.001 vs. unpaired and naive, ### *p*<0.001, #*p*<0.05 vs. saline. (A) Representative immunoblots shown in B.

A protein cross-linking assay [29] was used to compare the distribution of GluR1 and GluR2 after 90 CS-alone trials. Briefly, LA and BLA tissues were removed and cross-linked with BS^3^. BS^3^ selectively cross-links cell surface (S) proteins, forming high-molecular-weight aggregates. Intracellular (I) proteins are not modified and thus retain their normal molecular weight. A measure of total receptor subunit protein is obtained by summing S+I [30]. Analyses of GluR1 and GluR2 from naïve, unpaired, paired and 90 CS-alone trial rats are shown in figure 5B. The levels of surface expression of GluR1 and GluR2 relative to total (S/S+I) were significantly higher (Fig. 5B, left) (GluR1: F_(2,15)_ = 33.97, *p*<0.001; GluR2: F_(2,15)_ = 77.13, *p*<0.001) whereas intracellular GluR1 and GluR2 relative to total (I/S+I) were significantly lower in paired (Fig. 5B, right) than in naïve and unpaired rats. This conditioning-induced increase in surface expression of GluR1 and GluR2 was reversed by 90 CS-alone trials (*p*<0.001 vs. paired). Furthermore, the effect of 90 CS-alone trials could be blocked by MTEP in a dose-dependent manner (GluR1: F_(4,25)_ = 13.04, *p*<0.001; GluR2: F_(2,15)_ = 20.09, *p*<0.001).

To assess whether the decrease in surface receptors by prolonged extinction training resulted in changes of excitatory synaptic transmission, we measured the relative contribution of AMPA receptors and NMDA receptors to the EPSCs [31]. Amygdala slices were made from naïve, unpaired, paired, 30 CS-alone trials, 90 CS-alone trials and 90 CS-alone trials plus MTEP pretreatment rats 24 h after CS-alone trials. As shown in figure 6A, the AMPA/NMDA ratios were 1.59±0.10 (n = 6) and 1.57±0.30 (n = 6) in slices from the naïve and unpaired rats. The ratio was significantly higher in the paired rats (4.14±0.11, n = 6, F_(2,15)_ = 19.2, *p*<0.001) suggesting that fear conditioning persistently increased AMPA-mediated synaptic transmission. There was no difference in the AMPA/NMDA ratio between paired and 30 CS-alone trials rats (4.08±0.46, n = 6, *p*>0.5), suggesting that 30 CS-alone trials did not affect conditioning-induced increase in AMPA/NMDA ratio. However, in the 90 CS-alone trials-treated rats, AMPA/NMDA ratio (1.67±0.19, n = 6) was significantly lower than those of paired and 30 CS-alone trials rats (F_(2,15)_ = 12.25, *p*<0.001). There was no difference in AMPA/NMDA ratio between naïve, unpaired and the 90 CS rats (F_(2,15)_ = 0.6, *p*>0.5). These results suggest that 30 CS-alone trials failed to affect conditioning-induced increase in AMPA/NMDA ratio. Only by 90 CS-alone trials did extinction training reverse the increase. Moreover, the effect of 90 CS-alone trials was blocked by MTEP pretreatment (3.80±0.34, n = 6, *p*<0.001 vs. 90 CS-alone trials).

**Figure 6:** Effects of 90 CS-alone trials on conditioning-induced increases in AMPA/NMDA ratio and the expression of PSD-95 and SAP97. (A) Plot of AMPA/NMDA ratios in naïve, unpaired, paired, 30 CS, 90 CS and 90 CS+MTEP rats. ***p<0.001 vs. paired and 30 CS, ###*p*<0.001 vs. 90 CS. Scale: 50 ms, 100 pA. (B) Representative blots and mean ± SEM of PSD-95 immunoreactivity from rats that have been conditioned and 24 h later received 2–6 sessions of 15 presentations of light-alone trials. Lateral (LA) and basolateral (BLA) amygdala tissues were dissected out, and PSD-95 levels were determined by Western blot analysis. ***p<0.001, **p<0.01 vs. context control. (C and D) Representative blots and mean ± SEM of PSD-95 and SAP97 immunoreactivities from rats that received 90 CS-alone trials. LA and BLA tissues were dissected out at various time points after extinction training as indicated, and PSD-95 and SAP97 levels were determined by Western blot analysis. *p<0.05, **p<0.01, ***p<0.001 vs. context control.

Postsynaptic density-95 (PSD-95) is a scaffolding protein of the postsynaptic density, which interacts with GluR indirectly through stargazin and regulates GluR trafficking [32], [33]. We examined whether PSD-95 expression was altered after 90 CS-alone trials. Rats were conditioned and 24 h later received 2–6 sessions of CS-alone trials. Twenty-four hours later, LA and BLA tissues were dissected out and PSD-95 was determined by immunoblotting. As shown in figure 6B, conditioning-induced increase in PSD-95 was absent after 6 sessions of light-alone trials but was not affected by 2–4 sessions of trials. In the next experiment, rats were conditioned and 24 h later received 90 CS-alone trials. LA and BLA tissues were dissected out at 5, 10, 30, 60, 120, 240 and 360 min after 90 CS-alone trials. As shown in figure 6C, conditioning-induced increase in PSD-95 was reduced within 30 min after 90 CS-alone trials and abolished by 240 min (F_(7,40)_ = 11.98, *p*<0.001).

A PDZ-domain-containing protein SAP97 binds to GluR1 and traffics GluR1 into spines [34]. In the lateral amygdala, the coupling of A-kinase anchoring proteins (AKAPs) and protein kinase A (PKA) to GluR1 through SAP97 is essential for fear memory formation [35]. We examined whether SAP97 expression was altered after 90 CS trials. As shown in figure 6D, conditioning-induced increase in SAP97 was reduced at 120 min and abolished 240 min after 90 CS-alone trials (F_(7,40)_ = 6.89, *p*<0.001). In contrast to what was observed with 90 CS trials, 30 CS-alone trials failed to affect the level of PSD-95 (Fig. 6B).

### Effects of Disruption of AMPA Receptor Endocytosis on 90 CS Extinction

A synthetic peptide containing a short C-terminal sequence of GluR2 (_869_YKEGYNVYG_877_, GluR2_3Y_) has been shown to block LTD in the hippocampus and the nucleus accumbens [36], [37], and the extinction of learned fear [38], [39]. When fused to the cell membrane transduction domain of the HIV-1 Tat protein (Tat-GluR2_3Y_) creating a cell membrane permeable peptide, Tat-GluR2_3Y_ impairs extinction of fear memory. We performed behavioral assessment to determine whether Tat-GluR2_3Y_ influenced extinction. Rats received 10 light-shock pairings, followed next day by 90 CS-alone trials and percentage of fear-potentiated startle was measured 24 h after extinction training (Day 3, Test 1). Rats were given Tat-GluR2_3Y_ (_869_YKEGYNVYG_877_, 15 pmol in 0.8 µl saline per side, n = 7) or the control peptide Tat-GluR2_3A_ (_869_AKEGANVAG_877_, n = 6) bilateral to the amygdale 30 min before 90 CS alone trials. One rat with incorrect Tat-GluR2_3Y_ infusion placement was excluded from the analysis. Figure 7 shows that light-alone trial resulted in a reduction of startle potentiation in Tat-GluR2_3A_-treated rats and fear-potentiated startle was significantly less than that in the Tat-GluR2_3Y_ rats (t_(12)_ = 5.218, *p*<0.001). Rats were also tested at 6 days (Day 8, Test 2) and 13 days (Day 15, Test 3) after the extinction training and Tat-GluR2_3Y_ -treated rats showed higher level of startle potentiation than those of Tat-GluR2_3A_-treated rats.

**Figure 7:** Tat-GluR2_3Y_ blocks the effect of 90 CS-alone trials on extinction. (A) Rats received Tat-GluR2_3Y_ (15 pmol in 0.8 ml saline per side) or Tat- GluR2_3A_ (15 pmol in 0.8 ml saline per side) bilaterally into the amygdala 30 min before extinction training. Retention of memory was assessed 1 (Test 1), 6 (Day 8, Test 2) and 13 days (Day 15, Test 3) after extinction training. **p<0.01, ***p<0.001 vs. GluR2_3Y_. (B) Distribution of cannula tips in the amygdala from rats infused with Tat-GluR2_3Y_ (△) or Tat- GluR2_3A_ (▴).

## Discussion

The role of amygdala glutamate receptors in fear learning, fear-potentiated startle, and extinction has been proposed before [40]. Although mGluR5 in the lateral amygdala is implicated in the induction of long-term potentiation and the formation of fear memory [41], [42], its role in fear extinction in the limbic circuitry is not well established. A previous study has shown that intra-LA injection of CPCCOEt impaired extinction suggesting a contribution of mGluR1 [43]. In mGluR5 knock-out mice, acquisition of fear conditioning is partially impaired whereas the extinction of both contextual and auditory fear was completely abolished [44], [45]. Here we showed that prolonged extinction training resulted in an inability to retrieve memory at later times consistent with either a persistent or permanent inhibition of fear. An mGluR5 antagonist blocked the long-term inhibition whereas an mGluR1 antagonist was without effect. Furthermore we found that six- but not two-sessions of extinction training reversed conditioning-induced increase in surface expression of GluR1 and AMPA/NMDA ratio in an mGluR5-dependent manner. Finally, a GluR2-derivative peptide that blocked regulated AMPAR endocytosis reversed the inhibition of spontaneous recovery after prolonged extinction training. We interpret these data to suggest that prolonged extinction training results in an mGluR5-dependent long-term inhibition of fear recovery that may involve the degradation of the original memory. However, conditioned fear is usually measured by either fear-potentiated startle or freezing response. We used fear-potentiated startle paradigm and did not measure within-session extinction and extinction recall. Therefore, we could not differentiate between whether prolonged extinction makes it more likely that test sessions will produce more efficient and long lasting within-test-session extinction as opposed to prolonged extinction reducing spontaneous recovery directly.

Extensive extinction training induces greater reduction of conditioned response and reduced spontaneous recovery, implying that repeated extinction triggers the permanent depression of memory recovery [16], [46]. Once sufficient numbers of CS have been presented and extinction successfully induced, additional spaced presentations are more effective [16]. We used 6 sessions of 15 presentations of light-alone trials spaced by 10 min between each session and found that this protocol produced a greater reduction of fear-potentiated startle and less spontaneous recovery than that of 2 sessions. Loss of spontaneous recovery was not seen after application of the mGlu5 receptor antagonist MTEP.

Fragile X syndrome (FXS) is a monogenic developmental disorder associated with a complex neuropsychiatric phenotype [47]. FXS is caused by transcriptional silencing of the *FMR1* gene, which encodes fragile X mental retardation protein (FMRP)–an RNA-binding protein that regulates translation of its interacting mRNAs [28]. It has been proposed that exaggerated mGlu5-mediated signaling in the absence of FMRP plays a causal role in FXS. In FMRP-knockout animals, there is a marked increase of LTD in the hippocampus but no alterations in LTP [48]. The enhanced LTD in hippocampal neurons of knockout mice is a consequence of increased activity mediated by type 1 metabotropic glutamate receptors [49], [50]. In the present study, we first demonstrated that mGluR5 and new protein synthesis are involved in prolonged extinction training-induced inhibition of memory recovery in mice as seen in rats. Then using FMR1^−/−^ mice, we find reduced spontaneous recovery of fear memory after extinction training compared with wild type mice. These results further support the involvement of mGluR5 in the inhibition of spontaneous recovery of fear memory after prolonged extinction training.

It seems likely that our prolonged CS-alone extinction protocol that results in a long-term inhibition of spontaneous recovery acts through one of two mechanisms. First, it could be the protocol enhances consolidation of extinction memory. Alternatively, the loss of spontaneous recovery could be the consequence of unlearning. Notably, conditioning-induced increase in GluR1 was reversed after the prolonged CS-alone trials. Consistent with the latter hypothesis, inhibition of AMPA receptor endocytosis in the amygdala restored spontaneous recovery suggesting that extinction might be mediated by degradation of the original memory. It is conceivable that prolonged extinction training results in a large amount of glutamate release, which acts on perisynaptic mGluR5 leading to formation of inositol 1,4,5-trisphosphate (IP3) and diacyl glycerol. IP3 induced Ca^++^ release from internal stores may lead to the activation of calcineurin, whereupon calcineurin can cause the dephosphorylation of GluR1 Ser845 likely through the inactivation of phosphatase 1A inhibitor that may initiate endocytosis of GluR1 and GluR2 from the surface of neurons [51], [52]. Generally the signal transduction coupling mGluR5 to AMPAR endocytosis depends on the experimental conditions and the brain areas studied [53]. At cerebellar parallel fiber to Purkinje cell (PF-PC) synapses, mGluR5 activation is coupled to PLC activation, diacylglycerol production and protein kinase C (PKC) activation resulting in phosphorylation of GluR2 at Ser880 [54], [55] which reduces its affinity for the AMPAR scaffold GRIP leading to internalization of AMPAR. At hippocampal CA1 synapses, mGluR5 activation is coupled to protein synthesis [26] via PI3K-Akt mammalian target of the rapamycin (mTOR) [56] or ERK-MAPK [57] signaling pathways.

People suffering from phobias show impaired extinction of aversively conditioned responses [58], [59] and increased amygdala activity when exposed to traumatic stimuli [60], [61]. Therefore, methods of preventing the return of fear after exposure therapy may lead to more effective therapeutic interventions. In the present study, we have demonstrated that extended extinction leads to persistent attenuation of fear recovery via an mGluR5-dependent mechanism. These results may open a new avenue for the treatment of anxiety disorders.

## Materials and Methods

### Animals

All procedures were approved by the Institutional Animal Care and Use Committee of the College of Medicine, National Cheng-Kung University or Animals and animals were treated in compliance with the European Communities Council Directive (86/609/EEC). Animals were housed in cages of four rats or mice each in a temperature (24°C)-controlled animal colony; pelleted rat chow and water were available ad libitum. They were maintained on a 12∶12 light–dark cycle with lights on at 0700 h. All behavioral procedures took place during the animal light cycle. Male fmr1^−/−^ mice on a C57BL/6J genetic background [62] aged 10 to 11 weeks (P70 - 80) (fmr1^−/−^ ) were used, with wild-type littermates used as control group. Mice were genotyped by tail PCR as described by [62].

### Surgery

Male Sprague-Dawley rats (175–200 g), anesthetized with sodium pentobarbital (50 mg/kg, i.p.), were mounted on a stereotaxic apparatus and a cannula made of 22 gauge stainless steel tubing was implanted into the lateral (LA) or basolateral (BLA) amygdala [anteroposterior, –2.8 mm; mediolateral, ±4.5 mm; dorsoventral, –7.0 mm]. A 28 gauge dummy cannula was inserted into each cannula to prevent clogging. The rats were monitored and handled daily and were given 7 days to recover. MTEP (dissolved in saline. 10 µg/side for intra-amygdalar injection, and 2.5, 5 or 10 mg/kg for intraperitoneal injection) and CPCCOEt (dissolved in saline containing 45% 2-hydroxypropyl-β- cyclodextrin w/v. 5 mg/kg or 10 mg/kg for intraperitoneal injection) were purchased from Tocris Cookson Ltd (Northpoint, UK). Anisomycin (3 drops of Tween 80 in 2.5 ml of 7.5% DMSO in artificial CSF, and adjusted to pH 7.4 with NaOH. 62.5 µg/side for intra-amygdalar injection, and 100 mg/kg for intraperitoneal injection) was obtained from Sigma (St. Louis, Missouri). A TAT-conjugated peptide (GluR2_3Y_, YKEGYNVYG) designed to impair AMPA receptor endocytosis was dissolved in 0.9% NaCl and infused into the LA or BLA (15 pmol/side) bilaterally 30 min before extinction training. The control peptide had the sequence AKEGANVAG (GluR2_3A_). Dose was chosen with reference to Brebner et al. (2005) [35]. Drug was administered bilaterally to the amygdala in a volume of 0.5–0.8 µl at a rate of 0.1 µl/min. The infusion cannulas were left in place for 2 min before being withdrawn.

### Behavioral Apparatus and Procedures

Rats were trained and tested in a stabilimeter device. Behavioral experiments of fear conditioning and extinction training were performed in standard operant chamber (San Diego Instrument, San Diego). The acoustic startle stimulus was a 50 ms white-noise at the intensity of 95 dB. The visual CS was a 3.7 s light produced by an 8 W fluorescent bulb attached to the back of stabilimeter. The US was a 0.65 mA footshock with duration of 0.5 s. Rats were placed in the training/testing chamber for 10 min and returned to their home cages on three consecutive days to habituate them to the test chamber and to minimize the effect of contextual conditioning. Following two days, Rats were handled in the same chamber before fear conditioning for pre-exposure. During pre-exposure, baseline startle was measured on each of 2 d by presenting 30 startle stimuli at a 10 sec interstimulus interval (ISI). Rats having equivalent baseline mean startle amplitudes were then divided into separated matched groups. On the day of fear conditioning, the animal was brought to the room, allowed to habituate, and placed in the chamber as before. The CS–US pairing began after a 3 min acclimation period in the chamber.

#### Training

The rats were placed in the startle boxes and received 10 light-footshock pairings at an ITI of 2 min. Unpaired controls received the same number of light and footshock presentation, but in a pseudorandom fashion in which the US could occur at anytime except at 3.2 sec following the CS.

#### Extinction

The rats were returned to the stabilimeter 24 h after the training and given 2, 3, 4, 5, 6, 7 or 8 sessions of 15 presentations of the 3.7-s light with neither shock or a startle-elicited noise burst (light-alone trials). Each session was separated by 10 min with an ITI of 1 min.

#### Test

The rats were tested for fear-potentiated startle 1(Test 1), 6(Test 2) or 13(Test 3) days after Extinction training. This involved 10 startle-eliciting noise bursts presented alone (noise-alone trial) and 10 noise bursts presented 3.2 s after onset of the 3.7-s light (light-noise trials). The two trial types were presented in a balanced mixed order (ITI, 30 s). The percentage of fear-potentiated startle was computed as: [(startle amplitude on CS-noise minus noise-alone trials)/(noise-alone trials)]×100.

Fear conditioning for mice occurred in 30×24×21 cm operant chamber (Med Associates, St. Albons, VT). The chamber was cleaned with 75% ethanol before each mouse was trained or tested for contextual fear conditioning. On the first day, mice were placed in a context for 3 min and received a footshock every 60 sec for 5 times. After training, mice were randomly assigned to saline, MTEP 2.5 mg or MTEP 5 mg groups in which they received intraperitoneal injection of saline, MTEP 2.5 mg/kg or MTEP 5 mg/kg respectively one hour before extinction training. On day 2, mice were placed in the same context for 10 min without receiving footshock. The procedure was repeated 2 times with an interval of 30 min (Extinction training). Contextual freezing responses were measured on day 3 and day 8. The behavior of mice was recorded by video camera mounted above the conditioning chamber. Freezing was defined as the absence of any movement except for respiration and measured automatically using FreezeScan software. Freezing data are presented as percent time spent freezing.

### Whole-cell Patch-clamping Recordings for AMPA/NMDA Ratio

Whole-cell patch-clamp recordings from LA projection neurons were performed at ∼32°C in a superfusing chamber. Neurons were visualized with infrared video microscope using a 40× water immersion objective on an upright microscope. EPSCs were evoked at 0.03 Hz by extracellular stimulation of fibers emerging from the internal capsule which originate in the medial geniculate nucleus of the thalamus and project monosynaptically to the LA using a bipolar electrode. Patch electrodes were pulled from thick wall glass capillary (0.75 mm I.D., 1.5 mm O.D.) to a tip resistance of 3–5 MΩ. The composition of the internal solution was (in mM): Cs-gluconate 115, NaCl 5, EGTA 1, CaCl_2_, 0.3, MgCl_2_ 2, Na-ATP 5, Na-GTP 0.4, HEPES 10. The final pH of the internal solution was adjusted to 7.3 by adding 1 M KOH; the final osmolarity was adjusted to 280 mOsm by adding sucrose. Recordings were low-pass-filtered at 2.5–20 kHz and digitized at 5–50 kHz. The signal was monitored and recorded with an Axopatch 200B amplifier. On-line analysis and control of experimental acquisition is accomplished via a 586 (Intel)-based PC clone and a Digidata 1200 computer interface. AMPAR-mediated EPSC was evoked when the neurons were voltage-clamped at −70 mV whereas NMDAR-mediated EPSC was determined as current amplitude at 50 ms after peak EPSC amplitude at a holding potential of +40 mV. Bicuculline (10 µM) was present in the perfusion solution. To avoid bias, data were collected from one cell per animal.

### Surface Biotinylation of AMPA Receptor GluR1/R2 Subunits

Brain slices containing only LA and BLA were placed on ice and washed twice with ice-cold ACSF. The slices were then incubated with ACSF containing 0.5 mg/ml Sulfo -NHS- LC- Biotin (Pierce Chemical Co., Rockford, IL) for 1 h on ice. Next, the slices were rinsed in ACSF and then sonicated briefly in homogenizing buffer (1% Triton X-100, 0.1% SDS, 50 mM Tris-HCl, pH 7.5, 0.3 M sucrose, 5 mM EDTA, 2 mM sodium pyrophosphate, 1 mM sodium orthovanadate, 1 mM phenylmethylsulfonyl fluoride (PMSF), 20 µg/ml leupeptin, and 4 µg/ml aprotinin). After sonication, the samples were centrifuged at 14000 rpm for 30 min at 4°C and the supernatant was obtained. Protein concentration in the soluble fraction was then measured using a Bradford assay, with bovine serum albumin as the standard. Biotinylated protein (400 µg) from the supernatant was precipitated with 50 µl of 50% Neutravidin agarose (Pierce Chemical Co.) for 16 h at 4°C and washed 4 times with homogenizing buffer. Bound protein was re-suspended in 4 µl of SDS sample buffer and boiled. Biotinylated protein was resolved in 8.5% SDS-polyacrylamide gels, blotted electrophoretically to PVDF membrane, and blocked overnight in TBS buffer containing 5% non-fatty milk. Surface GluR1, GluR2 receptors and pan-cadherin (surface protein control) were detected by a biotinylation assay, followed by Western blot analysis that used either a GluR1 (1∶4000, Millipore), GluR2 (1∶5000, Millipore) or pan-cadherin (1∶2500; Sigma) antibodies, followed by HRP-conjugated secondary antibody for 1 hr. Other membranes were incubated overnight with PSD-95 (1∶10,000, Millipore), SAP97 (1∶5,000, Stressgen, Victoria, BC, Canada) and Actin (1∶10,000, Millipore). An enhanced chemiluminescence kit was used for detection. Western blots were developed in the linear range used for densitometry. GluR1 and GluR2 levels in the conditioned animals were expressed as a percentage of those in naïve controls without receiving light-shock pairings.

### Synaptoneurosome Preparation

Brain slices containing only LA and BLA were homogenized in 70 µl of ice-cold lysis buffer in an Eppendorf tube. The buffer consisted of 118.5 mM NaC1, 4.7 mM KC1, 1.18 mM MgSO_4_, 2.5 mM CaCl_2_, 1.l8 mM KH_2_PO_4_, 24.9 mM NaHCO_3_, 10 mM dextrose, 10 µg/ml adenosine deaminase, pH adjusted to 7.4 by bubbling with 95% O_2_+5% CO_2_. Proteinase inhibitors (0.0l mg/ml leupeptin, 0.005 mg/ml pepstatin A, 0.l mg/ml aprotinin and 5 mM Benzamide) were included in the buffer to minimize proteolysis. The homogenate was diluted with 350 µl of additional ice-cold lysis buffer. This mixture was loaded into a l-m1 tuberculin syringe attached to a 13-mm diameter Millipore syringe filter holder. The diluted filtrate was forced over three layers of nylon (Tetko, 100 µm pores) pre-wetted with 150 µl of lysis buffer, and collected in a 1.5 m1 Eppendorf tube. The nylon-pre-filtered mixture was loaded into another 1 ml tuberculin syringe and forced through a pre-wetted 5 µm Millipore nitrocellulose filter. The homogenate was kept ice cold at all times to minimize proteolysis. The filtered particulate was then spun at l000×g for l5 min at 4°C. The supernatant was removed, and the pellet (synaptoneurosome) was re-suspended in 80 µl of lysis buffer for Western blot analysis.

### Surface Receptor Cross-linking with bis(sulfosuccinimidyl)suberate

Surface and intracellular GluR1 and GluR2 levels were determined with a protein cross-linking assay. After conditioning or extinction training, rats were decapitated, brains were removed rapidly. Slices were added to Eppendorf tubes containing ice-cold artificial CSF spiked with 2 mM bis(sulfosuccinimidyl)suberate (BS3; Pierce Biotechnology, Rockford, IL). Incubation with gentle agitation proceeded for 15 min at 4°C. Crosslinking was terminated by quenching the reaction with 100 mM glycine (10 min at 4°C). The slices were pelleted by brief centrifugation, and the supernatant was discarded. Pellets were resuspended in ice-cold lysis buffer containing protease and phosphatase inhibitors [1% Triton X-100, 0.1% SDS, 50 mM Tris-HCl, pH 7.5, 0.3 M sucrose, 5 mM EDTA, 2 mM sodium pyrophosphate, 1 mM sodium orthovanadate, 1 mM phenylmethylsulfonyl fluoride (PMSF), 20 µg/ml leupeptin, and 4 µg/ml aprotinin, 1 µM microcystin-LF, 1 µM okadaic acid, 1×protease inhibitor mixture (EMD Biosciences, San Diego, CA), and 0.1% Nonidet P-40 (v/v)] and homogenized rapidly by sonicating for 10 s. A brief centrifugation was performed, and the supernatant fraction was used for further studies. Total protein concentration of the supernatant was determined by the Lowry method. Samples were aliquoted and stored at –80°C for future analysis.

### Histology

To identify cannula placements, animals received an overdose of pentobarbital (100 mg/kg) at the end of behavioral experiments. The brains were removed from the skull and fixed in buffered 4% paraformaldehyde for 48 h. Brains were sectioned with a microslicer (DTK-1000, Dosaka) and 40-μm-thick sections were stained for Nissl bodies.

### Data Analysis

All values in the text were mean±SEM. Differences among the groups were evaluated with one-way ANOVA followed by the Newman-Keuls *post hoc* tests. Single-factor ANOVA and Newman–Keuls *post hoc* comparisons were used to analyze the differences in AMPA/NMDA ratio among naïve, paired, unpaired and extinction groups. Unpaired *t* test, was used to analyze differences of startle reflex between drug-treated and vehicle control groups. The level of significance was *p*<0.05.
